The article "Synthesis and Optimization of Deesterified Acacia-Alginate Nanohydrogel for Amethopterin Delivery" was published in 2022. Journal: Bioinorg Chem Appl.

# Synthesis and Optimization of Deesterified Acacia-Alginate Nanohydrogel for Amethopterin Delivery

**DOI:** 10.1155/2022/7192919

**Published:** 2022-02-11

**Authors:** T. Sathish, N. Sabarirajan, S. Prasad Jones Christydass, S. Sivananthan, R. Kamalakannan, V. Vijayan, Prabhu Paramasivam

**Affiliations:** ^1^Department of Computer Science and Engineering, Saveetha School of Engineering, SIMATS, Chennai 602105, Tamil Nadu, India; ^2^Department of Mechanical Engineering, Chendhuran College of Engineering and Technology, Pudukkottai, Tamil Nadu, India; ^3^Department of Electrical and Electronics Engineering, K. Ramakrishnan College of Technology, Tiruchirapalli, Tamil Nadu, India; ^4^Department of Mechanical Engineering, K.Ramakrishnan College of Engineering, Samayapuram, Tiruchirapalli, Tamil Nadu, India; ^5^Department of Mechanical Engineering, M. Kumarasamy College of Engineering, Karur, Tamil Nadu, India; ^6^Department of Mechanical Engineering, College of Engineering and Technology, Mettu University, Metu 318, Ethiopia

## Abstract

Naturally obtained materials are preferable for the production of biomedicine in biomedical applications. *Acacia* gum is has recently become a hopeful one in the biomedicine production due to its excellent properties, namely, emulsifier, stabilizing mediator, suspending agent, etc. In this novel work, we synthesised and characterized the deesterified *Acacia* gum-alginate nanohydrogel (DEA-AG NPs) as a carrier for amethopterin (ATN) delivery. This combination is used in the drug effectiveness and tissue engineering. In this work, the Taguchi route is implemented for estimating of particle size and zeta potential (mV) through optimization. Following three parameters are considered for this work: DEA solution concentration (0.008, 0.016, 0.024, and 0.032 w/v %), alginate molecular weight (3, 6, 9, and 12 MW), and ATN/DEA ratio (1 : 4, 1 : 8, 1 : 12, and 1 : 16 w/w %). In particle size analysis and zeta potential analysis, the DEA solution concentration is highly influenced. Minimum particle size is found as 148.50 nm. Similarly, maximum zeta potential is identified as 29.5 mV.

## 1. Introduction

In the paramedical application the drug delivery is one of the fast-growing technologies for cancer nanotherapeutics. This technology considers nanoparticles as a controlled liberate reservoirs. Further, it can eradicate the restrictions of traditional cancer therapy [1]. The use of nanoparticles in cancer nanotherapeutics improves cellular systems, reduces side effects, and controls tumour development [2–4]. In cancer nanotherapeutics, some problems are raised due to the nanoparticle's size and stability in the physiological function.

Several nanoparticles are involved in the drug delivery system. Of all of them, the nanohydrogels are the most excellent and potential ones in the drug delivery system [5]. Better porous molecular formation, elevated hydrophilicity, and small size of nanogels are the considerable advantages of the nanohydrogels [6–8]. Nanohydrogels are effectively utilized in the drug delivery system both in active and passive conditions. The structural properties of nanohydrogels vary in medical and pharmaceutical applications, and the production of polymers is dependent on these structural properties [9–11]. The excellent biocompatibility of nanohydrogels based on water molecules is vastly used in medical and pharmaceutical appliances [12]. The massive characteristics of the nanoparticles and the high advantages of the hydrogel amalgamation are hopeful in the drug delivery system.

*Acacia* is one of the natural gums and has excellent properties, being highly soluble in water [13]. It controls the cholesterol levels and also assists to increase weight loss. Further improvement of the *Acacia* solubility nature was achieved by conducting deesterified *Acacia* (DFA). Continually, the DFA highly influenced to prepare the hydrogels with the addition of using positively charged polymers such as alginate [14–16]. Alginate is one of the anionic polymers. It possesses various properties such as high biocompatibility in nature, low toxicity, minimum cost, form a gentle gelation, bacteriostatic, and anticholesteremic [17, 18]. Alginate is one of the powder materials; it comprises sodium alginate, calcium sulphate, trisodium phosphate, diatomaceous earth, zinc oxide, and potassium titanium fluoride [19]. All these elements are mixed homogeneously in water to form a smooth gel to create a mold [20].

The present investigation focused on to prepare the *Acacia* gum-alginate nanoparticles (DEA-AG NPs) to hold the amethopterin (ATN) is produced by the coacervation method [21]. We hope that the DEA-AG nanohydrogel is one of the appropriate drug delivery systems in medical applications and tissue engineering [22]. Taguchi statistical analysis is incorporated into this experimental work to analyze the effects of parameters on the particle size and zeta potential (mV) of the nanohydrogel [23].

## 2. Materials and Methods

The *Acacia* gum is procured from Opera Chemisol India Private Limited, Chennai. Alginate powder (5 and 10 kDa) is purchased from the Kwality Chemicals Co., Valipalayam, Coimbatore. The remaining chemical items are procured from the Praxor Instruments and Scientific Co., Chennai. This experimental work considered the Taguchi analysis to optimize the parameters and also found the parameters' effects on the quality of the responses [24]. Orthogonal Array L16 is taken for conducting of parameters optimization in the preparation of nanaohydrogel and its properties [25]. ANOVA analysis is also conducted for evaluation of the parameter contribution in the particle size analysis as well as zeta potential analysis [26]. Minitab 18 statistical software is used for analyzing of parameters optimization and control of the S/N ratio in the experimental work. Three parameters and four levels are accounted for this experimental work, and it is presented in Table 1.

### 2.1. Experimental Procedure

In this work, the DEA is prepared by using the deesterification process of *Acacia* gum, as shown in Figure 1. The DEA is liquefied in the deionized water to obtain the different concentrations of DFA solution such as 0.008 w/v %, 0.016 w/v %, 0.024, w/v %, and 0.032 w/v %. Furthermore, different molecular weights (3, 6, 9, and 12 kDa) of the alginate powder are taken and dissolved in deionized water and 1 v/v % acetic acid combination solution [27–29]. After dissolving the alginate in the combined solution, it can be formed into the 0.4% (w/v) concentration of each solution effectively. Continually, the ATN solution is diluted with deionized water properly and receives the 2% (v/v) ATN solution [30–32]. The combination of ATN/DEA solution is achieved by the effect of stirring action using a magnetic stirrer. The blending of ATN-DEA solutions is considered at the ratios of 1 : 4, 1 : 8, 1 : 12, and 1 : 16 (w/w). The alginate solutions with various molecular weights are mixed with the ATN-DEA solution drop by drop. The stirring process is conducted for 20 min at atmospheric temperature for the prepared nanoparticles. Further a centrifuge process is conducted for 30 min at 18000 rpm [33]. Finally, the nanoparticles are precipitated.

The response values of particle size and zeta potential of the nanohydrogels are carried out by using of DLS (sizing), M3-PALS (zeta potential) equipment [34]. Initially, the precipitated nanohydrogel was dispersed in 1 ml of deionized water and all the readings were taken by using a 4 mW HeNe laser of 633 nm wavelength at 25°C. Finally, the consideration of the L16 array all the experiments are conducted.

## 3. Results and Discussion

Table 2 presents the entire experimental summary and output response of the particle size analysis and zeta potential analysis. The minimum particle size was recorded as 148.50 nm by the influence of 0.008 w/v% DEA solution concentration, 3 molecular weight of alginate, and 1 : 4 of w/w % ATN/DEA ratio. On the contrary, the maximum particle size was registered as 439.04 nm. In the zeta potential analysis, the maximum zeta potential was observed as 29.5 mV by involving of 0.032 w/v% DEA solution concentration, 3 molecular weight of alginate, and 1 : 16 of w/w % ATN/DEA ratio. The minimum zeta potential was observed as 20.5 mV.

### 3.1. Particle Size Analysis

Table 3 is the output of Taguchi analysis in which the DEA solution concentration is found to be better at level 1 as it offers a smaller mean particle size of 193.8 nm. In the case of alginate molecular weight, level three was the level that offered a minimum average particle size of 256.9 nm. For the ATN/DEA ratio factor, level 1 was found to be better as it offered a minimum mean particle size of 250.7 nm.

From Table 4, it is understood that the higher the signal (favourable response), the better. Table 4 also contains the output of Taguchi analysis in terms of signal-to-noise ratio. The factor DEA solution concentration was found to be better at level 1 as it offered a high signal-to-noise ratio of (−45.59) for the minimum particle size. In the case of alginate molecular weight, level three was found to be better as it offered a high signal-to-noise ratio of (−47.87) for the minimum particle size. For the ATN/DEA ratio factor, level 1 was found to be better as it offered a high signal-to-noise ratio of (−47.44) for the minimum particle size.

Figure 2 illustrates the main effects plot for mean and the S/N ratio of the particle size response.  Figure 2(a) shows the graphical representation of Table 3 (mean particle size responses), and Figure 2(b) demonstrates the graphical representation of Table 4 (favourable chances signal-to-noise ratio). The purpose of this graph is to exhibit the optimal process factors which support the research objective. This analysis aims to reduce the average particle size.  Figure 2(a) for the factor a DEA solution concentration level 1 (0.008) shows the minimum mean particle size response. Similarly, Figure 2(b) shows the maximum favourable chances (signal to noise ratio) at level 1 which is 0.008 w/v%. Hence, it is concluded that for the factor, a DEA solution concentration of 0.008 w/v% is optimal. Similarly, for the factor of alginate molecular weight, level 3 is found optimal, as Figures 2(a) and 2(b) show minimal mean particle size and maximum favourable chance (S/N ratio) at level 3 as 9 MW, respectively, and for the factor ATN/DEA ratio, the graphs at Figure 2(a) show minimum average particle size at level 1 as well as Figure 2(b) also indicates a higher signal-to-noise ratio at level 1 as 1 : 4 w/w %. Hence, the optimal process parameters or optimal input factors for obtaining the minimal mean particle size are 0.008 w/v% DEA solution concentration, 9 MW alginate, and a 1 : 4 of w/w % ATN/DEA ratio.

Minimum particle size was observed by the influence of 0.008 w/v% of DEA solution concentration, further increasing of DEA solution concentration the particle size also increased. A minimum level of alginate (MW) produced a maximum particle size; 9 MW of alginate offered a minimum particle size. In the ATN/DEA ratio parameter analysis, the minimum particle size was observed by the influence of a 1 : 4 ratio of ATN/DEA. All the data points were scattered uniformly and within the limit it was clearly exposed in the probability plot, as shown in Figure 3. In this experimental work, the chosen parameters of the acacia-alginate nanohydrogel for amethopterin delivery and the executed statistical model were appropriate ones.

Table 5 presents the ANOVA analysis for particle size; in this analysis, we point out the parameter contribution based on the *F* value. Among the three parameters, a higher contribution of 55.16% was observed by the influence of DEA solution concentration followed by 23.55% of the ATN/DEA ratio and 8.33% of alginate molecular weight. It is clearly noted that the DEA solution concentration changed the results of the particle size. *P* value of the all parameters were significantly sufficient, it can be noted that the *P* values were less than 0.05.

### 3.2. Regression Equation

Size (nm) = 299.8–106.1 DEA solution concentration (w/v%) 0.008 + 18.8 DEA solution concentration (w/v %) 0.016–1.7 DEA solution concentration (w/v %) 0.024 + 88.9 DEA solution concentration (w/v %) 0.032 + 25.1 alginate molecular weight (MW) 3 + 21.6 alginate molecular weight (MW) 6–43.0 alginate molecular weight (MW) 9–3.7 alginate molecular weight (MW) 12–49.2 ATN/DEA ratio (w/w %) 1 : 4–18.2 ATN/DEA ratio (w/w %) 1 : 8 + 74.4 ATN/DEA ratio (w/w %) 1 : 12–7.0 ATN/DEA ratio (w/w %) 1 : 16.

Figure 4 represents the correlations of two parameters' influence with the assist of a 3D trajectory plot.  Figure 4(a) illustrates the relations between DEA solution concentration and alginate molecular weight. From this analysis, the minimum particle size was observed by involving 0.008 w/v% DEA solution concentration and 3 molecular weights of alginate.  Figure 4(b) presents the correlations of alginate molecular weight and ATN/DEA ratio, minimum particle size was observed by the influence of 3 MW of alginate and a 1 : 4 ATN/DEA ratio.  Figure 4(c) illustrates the correlation between the ATN/DEA ratio and DEA solution concentrations. ATN/DEA ratio of 1 : 4 and 0.008 w/v% DEA solution concentration offered the minimum particle size.

### 3.3. Zeta Potential Analysis

Tables 6 and 7 represent the mean and S/N ratio of the zeta potential analysis. In this analysis, the DEA solution concentration was extremely influenced by the ATN/DEA ratio and alginate molecular weight.

Table 6 shows the output of Taguchi analysis for optimizing the process factors for maximizing zeta potential response. In Table 6, level 4 was found optimal for the DEA solution concentration as it offered a maximum mean particle size of 27.42 mV. In the case of alginate molecular weight, level 4 was the level that offered a higher average zeta potential response of 26.73 mV. For the ATN/DEA ratio factor, level 3 was found to be better as it offered a maximum mean zeta potential response of 27.63 mV.

It can be understood from Table 7 that the higher the signal (favourable response), the better. Table 4 also shows the output of Taguchi analysis in terms of signal-to-noise ratio. The factor DEA solution concentration was found to be better at level 4 as it offered a high signal-to-noise ratio of (28.75) for maximum zeta potential. In the case of alginate molecular weight, level 4 was found to be better as it offered a high signal-to-noise ratio of (28.53) for maximum zeta potential. For the ATN/DEA ratio factor, level 3 was found to be better as it offered a high signal-to-noise ratio of (28.81) for maximum zeta potential.

Optimal parameters of the zeta potential analysis were achieved as the following: 0.032 w/v% DEA solution concentration, 12 molecular weight of alginate, and 1 : 12 of w/w % ATN/DEA ratio.

Figure 5 reveals the main effects plot for the means and S/N ratio of the zeta potential analysis. A higher DEA solution concentration (0.032 w/v %) offered maximum zeta potential values. DEA solution concentration increases the zeta potential values of the nanaohydrogel. Increasing of alginate molecular weight increases the zeta potential analysis.

Figure 5 demonstrates that the main effects plot for means and S/N ratio of the zeta potential response.  Figure 5(a) shows the graphical representation of Table 6 (mean zeta potential responses), and Figure 5(b) demonstrates the graphical representation of Table 7 (favourable chances Signal to Noise Ratio). The purpose of this graph is to exhibit the optimal process factors which support the research objective. This analysis aims to reduce the average zeta potential. In Figure 5(a) for the factor, a DEA solution concentration at level 4 (0.032) shows the maximum mean zeta potential response. Similarly, Figure 5(b) shows the maximum favourable chances (signal-to-noise ratio) at level 4 which is 0.032 w/v%. Hence, it is concluded that for the factor a DEA solution concentration 0.032 w/v% is optimal. Similarly, for the factor of alginate molecular weight, level 4 is found optimal as Figures 5(a) and 5(b) show maximum mean zeta potential and maximum favourable chance (S/N ratio) at level 4 as 12 MW, respectively, and for the factor ATN/DEA ratio, the graphs at Figure 5(a) show maximum average zeta potential at level 3 as well as Figure 5(b) also indicates a higher signal-to-noise ratio at level 3 as 1 : 16 w/w %. Hence, the optimal process parameters or optimal input factors for obtaining the maximum zeta potential are 0.032 w/v% DEA solution concentration, 12 MW molecular weight of alginate, and 1 : 16 of w/w % ATN/DEA ratio.

In the zeta potential analysis, all the data points were distributed evenly and within the limit, as shown in Figure 6. Based on the data points distribution, the selected parameters and the model were good ones.

Table 8 presents the parameters' contributions in the zeta potential analysis; influence of contribution was estimated by the *F* values. In this analysis, the DEA solution concentration was extremely influenced such as 30.33%, followed by the ATN/DEA ratio (28.24%) and alginate molecular weight (18.85%).

### 3.4. Regression Equation

Zeta Potential (mV) = 25.869–2.219 DEA solution concentration (w/v %) 0.008 + 0.806 DEA solution concentration (w/v %) 0.016–0.144 DEA solution concentration (w/v %) 0.024 + 1.556 DEA solution concentration (w/v %) 0.032 + 0.556 alginate molecular weight (MW) 3 + 0.506 alginate molecular weight (MW) 6–1.919 alginate molecular weight (MW) 9 + 0.856 alginate molecular weight (MW) 12–1.569 ATN/DEA ratio (w/w%) 1 : 4–1.069 ATN/DEA ratio (w/w%) 1 : 8 + 1.756 ATN/DEA ratio (w/w%) 1 : 12 + 0.881 ATN/DEA ratio (w/w%) 1 : 16.

Figure 7 illustrates the relationship of two parameters influence with the aid of heatmap plot analysis.  Figure 7(a) represents the associations between DEA solution concentration and alginate molecular weight. From this analysis, the maximum zeta potential occurred by involving 0.032 w/v% DEA solution concentration and 3 molecular weight of alginate.  Figure 7(b) reveals the correlations between alginate molecular weight and ATN/DEA ratio, from this correlation the maximum zeta potential was recorded by the influence of 3 MW of alginate and 1 : 16 ATN/DEA ratio.  Figure 7(c) demonstrates the connection between the ATN/DEA ratio and the DEA solution concentration. From the ATN/DEA ratio and DEA solution concentration, the maximum zeta potential was registered at 1 : 16 of ATN/DEA and 0.032 w/v% of DEA solution concentration.

Using three parameters and an optimization process, this experimental work was developed, helping the scientific progress of medicine preparation. A lot of technology was involved to prepare the medicine. This work was a novelty in preparing the nanohydrogel using *Acacia* gum-alginate for drug delivery of amethopterin in medicine production.

## 4. Conclusion

Deesterified of *Acacia* gum-alginate nanoparticles (DEA-AG NPs) for amethopterin (ATN) delivery was successfully carried out. The responses of particle size and zeta potential were analyzed, and the optimal parameters were obtained. Finally, the results of this experimental work were drawn as follows:

- From the particle size analysis, the minimum particle size was found as 148.50 nm by the influence of 0.008 w/v% DEA solution concentration, 3 molecular weight of alginate, and 1 : 4 of w/w % ATN/DEA ratio. Similarly, in the zeta potential analysis, the maximum zeta potential was recorded as 29.5 mV by relating 0.032 w/v% DEA solution concentration, 3 molecular weight of alginate, and 1 : 16 w/w % ATN/DEA ratio.
- In the particle size analysis, the optimal parameters were found as 0.008 w/v% DEA solution concentration, 9 molecular weight of alginate, and 1 : 4 of w/w % ATN/DEA ratio. On the other hand, the optimal parameters of zeta potential analysis were obtained as 0.032 w/v% DEA solution concentration, 12 molecular weight of alginate, and 1 : 12 of w/w % ATN/DEA ratio.
- In the particle size analysis, elevated contributions such as 55.16% were recorded by the influence of DEA solution concentration followed by 23.55% of ATN/DEA ratio and 8.33% of alginate molecular weight. Similarly, in the zeta potential analysis, the DEA solution concentration was highly influenced such as 30.33%, followed by the ATN/DEA ratio (28.24%) and alginate molecular weight (18.85%).
- Both analyses, such as particle size and zeta potential, showed that the DEA solution concentration was highly influenced by the other two parameters.
- This research can be extended for fine tuning of this optimal solution by further characterization with the use of morphological analysis (TEM/SEM), differential scan calorimetry, swelling, degradation, and porosity of the hydrogel.

## Figures and Tables

**Figure 1:** Flow process of acacia-alginate nanohydrogel formation.

**Figure 2:** Main effects plot for (a) mean of particle size and (b) S/N ratio of particle size.

**Figure 3:** Probability plot for particle size.

**Figure 4:** 3D trajectory plot analysis for particle size effects with the combination of factors: (a) DEA solution concentration and alginate molecular weight, (b) alginate molecular weight and ATN/DEA ratio, and (c) ATN/DEA ratio and DEA solution concentration.

**Figure 5:** Main effects plot for (a) mean of zeta potential and (b) S/N ratio of zeta potential.

**Figure 6:** Probability plot for zeta potential.

**Figure 7:** Heatmap plot analysis for zeta potential effects with the combination of factors: (a) DEA solution concentration and alginate molecular weight, (b) alginate molecular weight and ATN/DEA ratio, and (c) ATN/DEA ratio and DEA solution concentration.

**Table 1:** Process parameters and their levels for Taguchi L16 experimental design.

S. no.	Parameters	Level 1	Level 2	Level 3	Levels 4
1	DEA solution concentration (w/v %)	0.008	0.016	0.024	0.032
2	Alginate molecular weight (MW)	3	6	9	12
3	ATN/DEA ratio (w/w %)	1 : 4	1 : 8	1 : 12	1 : 16

**Table 2:** Experimental process parameters and response summary of nanohydrogel preparation.

Exp. runs	DEA solution concentration (w/v %)	Alginate molecular weight (MW)	ATN/DEA ratio (w/w %)	Particle size (nm)	Zeta potential (mV)	S/N ratio of size	S/N ratio of zeta potential
1	0.008	3	1 : 4	148.50	20.5	43.4345	26.2351
2	0.008	6	1 : 8	180.64	22.3	45.1363	26.9661
3	0.008	9	1 : 12	250.70	24.6	47.9831	27.8187
4	0.008	12	1 : 16	195.28	27.2	45.8132	28.6914
5	0.016	3	1 : 8	300.12	26.8	49.5459	28.5627
6	0.016	6	1 : 4	354.17	27.9	50.9842	28.9121
7	0.016	9	1 : 16	211.34	23.6	46.4996	27.4582
8	0.016	12	1 : 12	408.97	28.4	52.2338	29.0664
9	0.024	3	1 : 12	412.07	28.9	52.2994	29.2180
10	0.024	6	1 : 16	325.78	26.7	50.2585	28.5302
11	0.024	9	1 : 4	187.34	22.4	45.4526	27.0050
12	0.024	12	1 : 8	267.58	24.9	48.5491	27.9240
13	0.032	3	1 : 16	439.04	29.5	52.8501	29.3964
14	0.032	6	1 : 12	425.18	28.6	52.5715	29.1273
15	0.032	9	1 : 8	378.19	25.2	51.5542	28.0280
16	0.032	12	1 : 4	312.67	26.4	49.9017	28.4321

**Table 3:** Mean particle size responses with respect to process parameters and their levels.

Level	DEA solution concentration (w/v)	Alginate molecular weight (MW)	ATN/DEA ratio (w/w %)
1	193.8	324.9	250.7
2	318.6	321.4	281.6
3	298.2	256.9	374.2
4	388.8	296.1	292.9
Delta	195.0	68.0	123.6
Rank	1	3	2

**Table 4:** Signal-to-noise ratio for particle size responses with respect to process parameters and their levels, the smaller the better.

Level	DEA solution concentration (w/v %)	Alginate molecular weight (MW)	ATN/DEA ratio (w/w %)
1	−45.59	−49.53	−47.44
2	−49.82	−49.74	−48.70
3	−49.14	−47.87	−51.27
4	−51.72	−49.12	−48.86
Delta	6.13	1.87	3.83
Rank	1	3	2

**Table 5:** Analysis of variance for particle size.

Source	DF	Seq SS	Contribution (%)	Adj SS	Adj MS	*F* value	*P* value
DEA solution concentration (w/v %)	3	78055	55.16	78055	26018	8.53	0.014
Alginate molecular weight (MW)	3	11818	8.35	11818	3939	1.29	0.030
ATN/DEA ratio (w/w %)	3	33327	23.55	33327	11109	3.64	0.023
Error	6	18308	12.94	18308	3051		
Total	15	141509	100.00				

**Table 6:** Mean of zeta potential responses with respect to process parameters and their levels.

Level	DEA solution concentration (w/v %)	Alginate molecular weight (MW)	ATN/DEA ratio (w/w %)
1	23.65	26.42	24.30
2	26.68	26.38	24.80
3	25.73	23.95	27.63
4	27.42	26.73	26.75
Delta	3.77	2.78	3.33
Rank	1	3	2

**Table 7:** Signal-to-noise ratio of zeta potential responses with respect to process parameters and their levels, the larger the better.

Level	DEA solution concentration (w/v %)	Alginate molecular weight (MW)	ATN/DEA ratio (w/w %)
1	27.43	28.35	27.65
2	28.50	28.38	27.87
3	28.17	27.58	28.81
4	28.75	28.53	28.52
Delta	1.32	0.95	1.16
Rank	1	3	2

**Table 8:** Analysis of variance for zeta potential.

Source	DF	Seq SS	Contribution (%)	Adj SS	Adj MS	*F* value	*P* value
DEA solution concentration (w/v %)	3	32.06	30.33	32.06	10.687	2.69	0.010
Alginate molecular weight (MW)	3	19.92	18.85	19.92	6.641	1.67	0.021
ATN/DEA ratio (w/w%)	3	29.86	28.24	29.86	9.952	2.50	0.046
Error	6	23.87	22.58	23.87	3.979		
Total	15	105.71	100.00				

## Data Availability

The data used to support the findings of this study are included in the article. Should further data or information be required, these are available from the corresponding author upon request.
